The article "A Comparative Study of Text Genres in English-Chinese Translation Effects Based on Deep Learning LSTM" was published in 2022. Journal: Comput Math Methods Med.

# A Comparative Study of Text Genres in English-Chinese Translation Effects Based on Deep Learning LSTM

**DOI:** 10.1155/2022/7068406

**Published:** 2022-06-02

**Authors:** Xiaoda Zhao, Xiaoyan Jin

**Affiliations:** Northeast Normal University, Changchun, 130024 Jilin, China

## Abstract

In recent years, neural network-based English-Chinese translation models have gradually supplanted traditional translation methods. The neural translation model primarily models the entire translation process using the “encoder-attention-decoder” structure. Simultaneously, grammar knowledge is essential for translation, as it aids in the grammatical representation of word sequences and reduces grammatical errors. The focus of this article is on two major studies on attention mechanisms and grammatical knowledge, which will be used to carry out the following two studies. Firstly, in view of the existing neural network structure to build translation model caused by long distance dependent on long-distance information lost in the delivery, leading to problems in terms of the translation effect which is not ideal, put forward a kind of embedded attention long short-term memory (LSTM) network translation model. Secondly, in view of the lack of grammatical prior knowledge in translation models, a method is proposed to integrate grammatical information into translation models as prior knowledge. Finally, the proposed model is simulated on the IWSLT2019 dataset. The results show that the proposed model has a better representation of source language context information than the existing translation model based on the standard LSTM model.

## 1. Introduction

It has been more than 60 years since the world's first machine translation system came out in 1954. At the same time, machine translation has gone through the flourishing situation of flourishing flowers and thriving competition, as well as the depression and silence of all sorts. The development paradigm of the mainstream machine translation technology has evolved from a rule-based approach to a statistical approach and then to today's neural network approach. Machine translation has also made its way out of the lab and into people's daily lives, addressing cross-language communication needs such as reading, meeting, travelling, and shopping [1]. Since 2013, the nerve machine translation because of the complicated characteristics of the project does not need to design a model that is concise and effective to get the favor of the researchers and developers, and parallel computing, graphics processors, and the wide application of big data in academia and industry quickly raised a hot wave nerve of machine translation research and development and advanced machine translation stride forward in the direction of practical application and commercialization.

The article "A Comparative Study of Text Genres in English-Chinese Translation Effects Based on Deep Learning LSTM" was published in 2022. Journal: Comput Math Methods Med.

Machine translation has both theoretical value and practical value and has experienced considerable development since its inception. Machine translation based on the neural network model has the following advantages:

1. End-to-end learning does not depend on too many prior assumptions. Phrase-based models, for example, assume that both source and target languages are sliced into sequences of phrases, with some alignment between them [2]. This hypothesis has both advantages and disadvantages. On the one hand, it draws lessons from the relevant concepts of linguistics and helps to integrate the model into human prior knowledge. On the other hand, the more assumptions there are the more constrained the model is. If the assumptions are correct, the model can describe the problem well. But if the assumptions are wrong, the model can be biased. Deep learning does not rely on prior knowledge, nor does it require the manual design of features. The model learns directly from the mapping of input and output (end-to-end learning), which also avoids possible deviations caused by assumptions to a certain extent
2. The continuous space model of neural network has a stronger representation ability. A basic problem in machine translation is how to represent a sentence [3]. The discrete lexical representation is replaced with a distributed representation of the space of real numbers, and the complete sentence can be expressed as a vector of real numbers

One of the important ideas is to integrate linguistic knowledge into a neural network to improve system performance and translation quality. Throughout the history of machine translation, linguistic knowledge has been playing an irreplaceable role. In particular, in the early stage, when the rule-based approach is dominant, from semantic analysis to target language generation, including the design of translation rules, all are guided by the internal connection of languages. The development of morphology, syntax, and semantics has been providing fuel for rule-based machine translation technology [4]. In the golden decade of statistical machine translation, there is use of hierarchical phrases to solve the problem of long-distance-dependent word translation and the use of sentence theory to solve the problem of short intonation order of target language. The language has serialization features; the source language and target language are strings, making the model simple, no longer needing the segmentation of complex, alignment, and sequence, such as processing, but at the same time also makes many important information losses in the process of linguistics [5]. The integration of the neural machine translation model, with it, can ease the predicament of inherent in the nerve machine translation, improve the nerve machine translation model, and further enhance the quality of translation.

The article "A Comparative Study of Text Genres in English-Chinese Translation Effects Based on Deep Learning LSTM" was published in 2022. Journal: Comput Math Methods Med.

The paper's organization paragraph is as follows. The related work is presented in Section 2.  Section 3 analyzes the algorithm design of the proposed work.  Section 4 discusses the experiments and results. Finally, in Section 5, the research work is concluded.

## 2. Related Works

In this chapter, we define the traditional machine translation and neural machine translation in detail.

### 2.1. Traditional Machine Translation

As early as the 17th century, attempts were made to overcome the human language barrier by using robotic dictionaries, similar to the use of quick lexicography devices like Kuai to solve communication problems between speakers of different languages [6]. In the 1930s, French engineer Archovny and former Soviet inventor Troyansky, respectively, designed and implemented the machine translation model system, which can be regarded as the prototype of machine translation. In 1954, Georgetown University and IBM jointly developed the first machine translation system in human history. Since then, with the joint efforts of colleges and universities, research institutes, enterprises, and even individuals, new technologies have emerged, new paradigms have emerged, and new systems have come into being. The level of machine translation has become higher and higher, and the quality of translation has become better and better, approaching or even surpassing the level of human beings in some specific fields [7]. In the development of machine translation, different machine translation technologies in different historical periods occupy the mainstream position.

Generally, rule-based machine translation can choose to transform at different levels, as shown in Figure 1. A complete rule-based machine translation process consists of the following steps:

1. Source language analysis: from shallow to deep, it can include morphological analysis, syntactic analysis, and semantic analysis, and ideally, it can become an intermediate language [8]. The segmentation and labeling rules for morphological analysis, the phrase structure rules for syntactic analysis, and the logical semantic rules for semantic analysis all need to be designed manually
2. Conversion from the source language to the target language: the bilingual dictionary is constructed, and the transformation mapping rules are designed on the basis of which, the transformation process is completed by replacing source language units with target language units and replacing source language structures with target language structures
3. Target language generation: according to the characteristics of the target language, the generation rules of the target language are designed

In the translation of low-resource languages and national languages with a short corpus, the rule-based method still provides unrivalled benefits. At present, some mature commercial machine translation systems on the market, especially those in certain limited fields, are based on rules. The advantage of the rule-based approach is that it is intuitive and can directly express linguistic knowledge. The degree of refinement of rules can be changed according to needs, and the rules with strong generalization ability can be used, and the rules with fine description ability can be used. It is easy to deal with complex structures and deep understanding; the system is highly adaptable and does not depend on a specific corpus [9]. However, the disadvantages are also obvious. The construction of rules relies too much on linguists, which is highly subjective and sometimes does not conform to the linguistic facts. The coverage of rules is poor, especially the knowledge of fine granularity is difficult to be summarized comprehensively, and the statements beyond the description of rules cannot be processed. As the number of rules increases, the conflicts between rules become more serious. The rule base is usually limited to a specific system, which is expensive to develop and difficult to maintain.

The article "A Comparative Study of Text Genres in English-Chinese Translation Effects Based on Deep Learning LSTM" was published in 2022. Journal: Comput Math Methods Med.

Its basic idea is that it does not need to conduct deep linguistic analysis and does not need a large amount of artificial summarized linguistic knowledge, but uses the translated corpus in the past and carries out translation by analogy. It assumes that the same part of the source language corresponds to the same translation result and that, when the previously translated part appears again, the same translation result is most likely the correct result. The main knowledge source of the system is the bilingual-aligned translation instance library [10]. The three core problems of the case-based approach are the correct bilingual automatic alignment, the establishment of an effective instance matching mechanism, and the generation of translation corresponding to the source language sentence based on the retrieved instances. The key technique is similarity calculation. There are no manual rules, there is no deep language analysis, the system development cost is low, and the speed is fast. The knowledge learned from the corpus is objective and covered well. However, the system performance depends heavily on the corpus. With serious data sparsity problem, it is difficult to make use of coarse granularity, general knowledge, and other deficiencies.

The article "A Comparative Study of Text Genres in English-Chinese Translation Effects Based on Deep Learning LSTM" was published in 2022. Journal: Comput Math Methods Med.

Statistical machine translation studies the translation process, the word alignment, the phrase segmentation, short tone sequence, such as syntax tree as an implicit structure, with the help of the machine learning techniques, statistical analysis on massive parallel corpora, on the basis of learning from the characteristics of the translation rule, finally using the model of the learning to translate. The basic idea of this model is as follows. Firstly, phrase-to-phrase translation rules are extracted from the parallel corpus of bilingual sentence alignment. During translation, the source language sentences are divided into phrase sequences, and the target language phrase sequences are obtained by translation rules. Then, the sequence of target language phrases is sorted by using the reordering model to obtain the best target translation [11]. While the research focus is on syntactic-based statistical translation models, how to improve the disambiguation ability of the models by introducing deeper linguistic analysis, while avoiding errors caused by analysis, has become the main problem faced by statistical translation models. In general, a statistical machine translation system has the following advantages: no need to write rules manually, translation model can be directly trained by corpus; system development cycle is short, labor cost is low, system robustness is good; high interpretability of hidden structure; exponential structural spaces are processed by local features and dynamic programming [12]. However, statistical machine translation systems also have the following shortcomings: discrete representation brings serious data sparsity problems; difficulty dealing with long-distance dependencies.

### 2.2. Neural Machine Translation

Neural network, especially deep learning technology, is the latest research achievement in the field of artificial intelligence. It enables people to use machine processing to process information in a new way and method. In just three or four years, machine translation has surpassed statistical methods in most language translation, and since then, machine translation has entered a “new era.”

At the end of 2013, Kalchbrenner proposed an encoder-decoder structure that can be used for machine translation, which immediately attracted extensive attention in the academic world; Google neural machine translation uses the long and short memory model and attention mechanism of 8-layer encoder and 8-layer decoder, integrating the important achievements of deep learning research in recent years and advancing machine translation in engineering practice a big step forward [13]. In May 2017, Facebook announced neural machine translation that was nine times faster than Google's accuracy. In September DeepL, based in Cologne, Germany, said its neuromachine translation product had beaten systems from Google, Microsoft, and Facebook in blind tests. On March 14, 2018, Microsoft announced that its Chinese-English system has achieved human-level performance on the news test set, a universal news corpus, and is “comparable to humans.” Other tech giants are also getting into the act, with Amazon, IBM, NVIDIA, and SYSTRAN all investing in neural machine translation systems. In this area, China is not to be outdone. Baidu, Youdao, Tencent, and Sougou have also joined the arms race, deploying their own neuromachine translation products. On May 20, 2015, Baidu Translation officially launched its neural machine translation system, becoming the first truly practical neural machine translation (NMT) system in the world [14]. On May 24, 2018, the Ali Machine Intelligence natural language processing (NLP) translation team won 5 titles in the workshop on machine translation (WMT), an internationally recognized top machine translation competition.

The article "A Comparative Study of Text Genres in English-Chinese Translation Effects Based on Deep Learning LSTM" was published in 2022. Journal: Comput Math Methods Med.

As early as 2003, Bengio, the father of deep learning, Turing Prize winner, and professor at the University of Montreal in Canada, proposed to improve the language model by using a neural network to represent each word as a continuous and dense vector of real numbers, effectively alleviating the problem of data sparsity. Jacob of BBN, an American company, further proposed a neural network combined model on this basis, which improved the quality of machine translation by about 6%. They adopted an “encoder-decoder” framework, and the translation process is shown in Figure 2. In this new framework, the linear model of statistical machine translation is replaced by the nonlinear model of the neural network, especially the circular neural network which is good at processing historical information, and variable-length string structure is added [15]. As soon as it comes into being, it attracts widespread attention from the academic circle and soon sets off a wave of research.

In addition to poor interpretability, neuromachine translation currently has the following problems. First, it is difficult to deal with rare words and unknown words. Second, there is the phenomenon of “overtranslation” and “omission.” Third, the translation is not faithful. The root cause of these problems is the neural machine translation architecture itself [16]. One of the important ideas is to integrate linguistic knowledge into a neural network to improve system performance and translation quality. Throughout the history of machine translation, linguistic knowledge has been playing an irreplaceable role. The source language and target language have been serialized as a string, and this makes the model simple and does not need to go through complex segmentation, alignment, and sequence.

The article "A Comparative Study of Text Genres in English-Chinese Translation Effects Based on Deep Learning LSTM" was published in 2022. Journal: Comput Math Methods Med.

## 3. Algorithm Design

In this section, we studied the LSTM model, attention embedding model based on LSTM, and translation model combined with grammar dependence.

### 3.1. LSTM Model

LSTM solves the long order dependence problem in the recurrent neural network; its specific network structure is shown in Figure 3. In addition to input data *X* and hidden state *H*, the LSTM network structure also includes memory unit *C*, input gate *I*, output gate *O*, and forgetting gate *F* [17]. The core of the LSTM model is to delete or add information in the memory cell state through a threshold structure composed of a sigmoid network layer and point-by-point multiplier.

Assuming that there exists batch data *X*_*t*_ at time *t* with *n* sample numbers, vector *x*, hidden layer length *H*, hidden layer state *H*_*t*_ at time *T*, and hidden layer state *H*_*t*−1_ at the previous time, the forgetting gate at time *T* can be expressed as

(1) $$\begin{array}{c} f_{t}=\sigma \left(X_{t}W_{xf}+H_{t-1}W_{hf}+b_{f}\right), \end{array}$$

where *σ* represents the sigmoid function; *X*_*t*_ represents the weight parameters that can be learned, *H*_*t*_ represents the bias vector parameters, and its addition process adopts the broadcast data operation method. Second, determine the information the memory unit needs to hold. The sigmoid network layer is adopted to determine the value of the update, as shown in equation (2). The hyperbolic tangent function tanh layer is used to generate candidate values, as shown in equation (3).

(2) $$\begin{array}{c} i_{t}=\sigma \left(X_{t}W_{xi}+H_{t-1}W_{hi}+b_{i}\right), \end{array}$$

(3) $$\begin{array}{c} {\bar{C}}_{t}=\tanh\left(X_{t}W_{xc}+H_{t-1}W_{hc}+b_{c}\right). \end{array}$$

Then, the memory state is updated. Dot product operation is adopted to update the state, and information flow is controlled by forgetting gate and input gate, so the updated state can be obtained, as shown in

(4) $$\begin{array}{c} C_{t}=f_{t}\Theta C_{t-1}+i\Theta {\tilde{C}}_{t}. \end{array}$$

When the input gate is constantly close to 0 and the forgetting gate is always close to 1, the memory unit in the old state is stored to the present moment [18], according to the preceding formula. Therefore, the LSTM network can solve the problem of gradient disappearance in the circulating nerve. Finally, the sigmoid layer is used to determine the state of memory unit output by the output gate, as shown in

(5) $$\begin{array}{c} O_{t}=\sigma \left(X_{t}W_{xo}+H_{t-1}W_{ho}+b_{o}\right), \end{array}$$

(6) $$\begin{array}{c} H_{t}=O_{t}\Theta \tanh\left(C_{t}\right). \end{array}$$

According to the above formula, when the output gate is approximately 0, the memory unit retains the current information, and when the output gate outputs 1, the information will be transferred from the storage unit to the hidden layer.

The article "A Comparative Study of Text Genres in English-Chinese Translation Effects Based on Deep Learning LSTM" was published in 2022. Journal: Comput Math Methods Med.

### 3.2. Attention Embedding Model Based on LSTM

LSTM network model in the coding stage is fixed dimension, so it adopts the vector of the same dimension to encode the source language sequence of any length. However, in actual English machine translation, the English input sequence is an indefinite sequence, which leads to the problem that the model and the English input sequence cannot completely fit in the machine translation using the standard LSTM model, and thus, the translation effect is not ideal [19]. The LSTM translation model embedded with attentional mechanism is shown in Figure 4, including encoding source language, attentional mechanism assistance, and target language generation process.

The state calculation method of the next hidden layer at the target end of the model is the same as that of the LSTM decoder, as shown in

(7) $$\begin{array}{c} Z_{i}+1=\sigma \left(c_{i},u_{i},z_{i}\right), \end{array}$$

where *u*_*i*_ represents the *i*^th^ word in the sequence of target language; *c*_*i*_ represents the background vector of the word *i* [20]. Assume that the hidden layer state at the moment *j* of the encoder is *H*_*j*_, and its corresponding background vector can be calculated by

(8) $$\begin{array}{c} C_{i}=\overset{T}{\underset{j=1}{\sum }}a_{ij}h_{j}, \end{array}$$

where *a*_*ij*_ represents the weight, which can be calculated by

(9) $$\begin{array}{c} a_{ij}=\frac{\exp\left(e_{ij}\right)}{\sum_{k=1}^{T}\exp\left(e_{ik}\right)}, \end{array}$$

(10) $$\begin{array}{c} e_{ij}=a\left(z_{i},h_{j}\right), \end{array}$$

where *a* is a function used to measure the matching degree between the current hidden state *z*_*i*_ of the target language sequence and the hidden state *h*_*i*_ of the source language sequence, which can be calculated by

(11) $$\begin{array}{c} e_{ij}=v^{T}\tanh\left(W_{zZi}+W_{h}h_{j}\right), \end{array}$$

where *v*, *W*_*z*_, and *W*_*h*_ represent the model parameters to be learned.

### 3.3. Translation Model Combined with Grammar Dependence

In neural machine translation, the degree of intimacy between each word in the sentence not only helps build a better earth beneath context, richer to express the meaning of the sentence, but it also allows the attention mechanism of dependencies between the source term to be passed to the decoder, better modelling source translation corresponding relationship between words and target words. This chapter will introduce how to obtain grammar dependence, introduce a distance mechanism based on grammar dependence, and combine grammar dependence with attention to improve the ability of attention to model words and grammar (machine translation generally considered rare between source language and target language, such as between Chinese and English grammar structure difference, is not suitable to handle this difference easily leading to loss of grammatical information, understanding sentences lack precision caused by translation system, failed to express the context of the sentence, a syntax, morphology, word order-disorder, such as error phenomenon) [21]. It makes the translation difficult to understand. It is the most direct and effective way to deal with the difference in grammatical structure to attach grammatical information to neural machine translation as prior knowledge. The common methods include, for example, taking dependent labels as input features of words, linearizing dependency tree to obtain source dependent representation sequence, learning source-side dependency graph representation by potential graph parsing, and using source and target-side dependency tree to improve neural machine translation. These methods are all based on the linear structure neural network to linearize the representation of grammatical information and grammatical structure. However, excessively long linearized sequences will affect the training efficiency, while using shorter sequences will lose the grammatical information, making it difficult to make a good compromise choice.

The article "A Comparative Study of Text Genres in English-Chinese Translation Effects Based on Deep Learning LSTM" was published in 2022. Journal: Comput Math Methods Med.

The article is the relative word between the head word of a noun phrase and its determinate word, according to the Stanford-type dependency manual [22]. The adjective modifier in a noun phrase is any word or phrase used to modify the meaning of a noun phrase, according to the Stanford-type dependency manual. To summarize, modifiers and articles alter and limit nouns, respectively, and it is clear that the former has a bigger impact on the word it operates on than the latter. “Excellent” describes the subject of the sentence “watchmaker,” whereas “this” characterises the subject of the sentence “watchmaker” who “produced many gorgeous watches” for the following events. Through qualitative analysis, we can draw a preliminary conclusion: the degree of dependent grammatical intimacy between different parent-child or grandparent node pairs is different.

At the same time, though, grammatical distance can also describe how close dependent grammatical relationships are between words. However, at a higher level of granularity, notice that the grammatical distance between the contiguous words is defined as 1. In other words, the degree of dependence is defined as 1 by the two-word pairs that have a direct dependency relationship and then extends to any two-word pairs in the sentence [23]. However, it is difficult to accurately describe the degree of intimacy of dependence between different father-son pairs only by the grammatical distance, because their grammatical distance is 1. This shows two situations: one, we cannot get the contribution degree of different child nodes to the same parent node, as shown in the red and yellow boxes in Figure 5, and another, we cannot describe the syntactic dependence closeness degree of different parent-child pairs, as shown in the red and green boxes in Figure 5. In Figure 5, the basic grammatical distances between all contiguous word pairs are represented by blue numbers.

Although the transformation process of grammatical distance from qualitative to quantitative is easy to realize, quantification of all pairs of dependencies in the same degree will inevitably lead to inconsistency between the intimacy of the dependency relationship and the grammatical distance, and the corresponding noise information will be introduced. The concept of “grammar dependence degree” can accurately describe the degree of dependent grammar intimacy between different parent and child pairs and obtain the numerical dependent grammar relationship between parent and child pairs. In other words, it can obtain the contribution degree of different child nodes to the parent node in constructing a dependent grammar context.

## 4. Experiments

In this part, we study the dataset source and pretreatment, model experiment in detail.

### 4.1. Dataset Source and Pretreatment

In this study, data from the 2019 International Oral English and Translation Evaluation Competition with a relatively small scale were selected as the experimental dataset, including 220,000 Chinese-English parallel sentence pairs, 3 test sets, and 1 development pair. In this study, word segmentation was carried out for the data, and then, CBOW was used to vector the data.

Since the IWSLT2019 dataset contains Chinese and English parallel sentence pairs and the word segmentation methods in Chinese and English are different, the Chinese and English datasets are processed by word segmentation, respectively. For Chinese word segmentation, the word segmentation method based on statistics is adopted. Then, according to the credibility of the word, the threshold value is set to form the word-formation conditions and determine the word segmentation. For English word segmentation, because the basic constituent unit of English is a word, therefore, only according to the blank can be directly split. English stop words processing mainly include three steps, first in English uppercase to lowercase, and then the statement tail words and symbols on the blank space, finally, therefore, adopt the method of proper nouns, with statements generalization processing, has completed the English word segmentation processing digitally to quantify the language symbols; language symbols can be input model to carry on the training study. In this study, CBOW was used to vectored words. In our study, the BLEU value is still used as an indicator to evaluate the performance of translation models. The higher the BLEU value, the better the translation quality.

The article "A Comparative Study of Text Genres in English-Chinese Translation Effects Based on Deep Learning LSTM" was published in 2022. Journal: Comput Math Methods Med.

### 4.2. Model Experiment

The regular LSTM model and the embedded LSTM model were initially trained on the experimental dataset to test the performance of the proposed translation model, and the results are collected in Figures 6 and 7. As can be seen from Figure 6, the LSTM model of attention embedded began to stabilize after 80 training rounds, which may be due to the strong learning ability of the attention mechanism, which enabled the LSTM model to learn the corresponding expression of text in a short time and thus tended to stabilize in a relatively short time.

However, it can also be seen from Figure 7 that due to the absence of term information input as prior knowledge in the source language, the translation model cannot fully learn the corresponding relationship between terms at the source end and terms at the target end during training and can only translate simple terms correctly, so the translation effect for long terms is not good.

Then, the standard LSTM model and the LSTM model combined with syntactical prior knowledge were used to train the experimental dataset. The results are shown in Figures 8 and 9. But because of using only a simple identifier for the target side terms are identified, therefore, the training time is longer than that without any identifiers and shorter than that with multiple complex identifiers.

Furthermore, as shown in Figure 9, simple identifiers used to identify target-end terms as a group can help the translation model better incorporate terminology knowledge during training, allowing the model to learn the semantic relationship between target-end terms and source statements.

The baseline model is based on standard LSTM, and the comparison method is attention-embedded LSTM model and grammatical prior knowledge LSTM model. The experimental results of each model are shown in Tables 1 and 2. As shown in Table 1, the BLEU value is still used as the evaluation standard when comparing the results of data enhancement methods of LSTM, LSTM+Attention, and LSTM+Grammar models during dataset verification. It can be seen that the bilingual corpus generated by using the translation model combining attention mechanism and prior grammar knowledge proposed in this paper achieves higher translation indicators than the standard LSTM translation model and is superior to the single data enhancement method as well as no data enhancement method.

The article "A Comparative Study of Text Genres in English-Chinese Translation Effects Based on Deep Learning LSTM" was published in 2022. Journal: Comput Math Methods Med.

Then, the experimental results of the standard LSTM model, the attention-embedded LSTM model, and the LSTM model with syntactic prior knowledge are compared on the processed dataset. As shown in Table 2, the LSTM model combining grammatical prior knowledge has the best translation effect. However, the attention-embedded LSTM model also has a good effect on the parallel corpus after grammar correction, which verifies the necessity of grammar correction for pseudocorpus. Experimental results show that the neural translation model is more sensitive to the quality of the corpus, and certain grammatical errors do not affect the translation performance but enhance the robustness of the model encoder.

## 5. Conclusion

To complete the translation process from source to destination language, the neural translation system employs the “encoder-attention-decoder” framework. The attention mechanism, on the other hand, has some flaws and unsolved issues, and syntactic prior information is not taken into account in the general neural machine translation system. As a result, how to improve the attention mechanism, lower computational costs, learn the internal relationships in the sequence better, and capture more accurate and rich context information; and how to integrate rich grammar knowledge, better model the semantic and syntactic representation of word sequence, improve sentence context understanding, and reduce grammatical errors in translation, among other things. Therefore, the English-Chinese translation model based on LSTM attention embedding and the LSTM model combined with grammatical prior knowledge is proposed. The innovation lies in the introduction of attention mechanism and grammatical prior knowledge into the standard LSTM translation model to enhance the representation of source language context information, thus improving the performance of the translation model and translation quality. Compared with the standard LSTM model, the proposed translation model has better performance, better translation effect, and better text genre.

The article "A Comparative Study of Text Genres in English-Chinese Translation Effects Based on Deep Learning LSTM" was published in 2022. Journal: Comput Math Methods Med.

## Figures and Tables

**Figure 1:** Machine translation at different levels of transformation.

**Figure 2:** Encoder-decoder translation schematic diagram.

**Figure 3:** Schematic diagram of LSTM network structure.

**Figure 4:** LSTM translation model embedded with attention mechanism.

**Figure 5:** The basic grammatical distance between the connected word pairs in the dependency tree.

**Figure 6:** Epoch/BLEU variation diagram between LSTM and LSTM+Attention.

**Figure 7:** Sentence/BLEU variation diagram between LSTM and LSTM+Attention.

**Figure 8:** Epoch/BLEU variation diagram between LSTM and LSTM+Grammar.

**Figure 9:** Sentence/BLEU variation diagram between LSTM and LSTM+Grammar.

**Table 1:** Experimental results of data enhancement method.

Method	Model	Validation set	Test set
Standard	LSTM	17.60	17.10
	LSTM+Attention	19.50	18.40
	LSTM+Grammar	21.30	20.20

Data enhance	LSTM	19.20	18.60
	LSTM+Attention	21.70	20.90
	LSTM+Grammar	23.10	22.50

**Table 2:** Experimental results of data pretreatment method.

Data format	Model	Validation set	Test set
Standard	LSTM	18.40	16.80
	LSTM+Attention	20.30	17.50
	LSTM+Grammar	20.70	19.40

Vector	LSTM	20.80	19.20
	LSTM+Attention	22.40	21.30
	LSTM+Grammar	24.30	22.70

## Data Availability

The datasets used during the current study are available from the corresponding author on reasonable request.
